# Skin mechanical properties measured with skin elasticity measurement device in patients with lymphedema: Scoping review

**DOI:** 10.1111/srt.13861

**Published:** 2024-08-03

**Authors:** Yudai Fujimoto, Yoshimi Yuri, Hironari Tamiya

**Affiliations:** ^1^ Department of Rehabilitation Osaka International Cancer Institute Osaka Japan; ^2^ Graduate School of Health Sciences Morinomiya University of Medical Sciences Osaka Japan; ^3^ Department of Orthopaedic Surgery (Musculoskeletal Oncology Service) Osaka International Cancer Institute Osaka Japan

**Keywords:** Cutometer, distensibility, elasticity, International Society of Lymphedema, outcome, parameter

## Abstract

**Background:**

Skin conditions in patients with lymphedema have been identified according to changes in skin mechanical properties. The skin elasticity meter is a non‐invasive tool for measuring the mechanical properties of the skin; however, its potential use in patients with lymphedema has received little attention. This review aimed to provide an overview of studies measuring the skin mechanical properties of patients with lymphedema using a skin elasticity meter.

**Materials and methods:**

Search terms and synonyms related to lymphedema and skin mechanical property measurement using a skin elasticity meter were identified, and electronic databases containing articles in English were searched.

**Results:**

A total of 621 articles were retrieved, and four articles were analyzed after screening. Despite this research subject receiving increasing attention, no consensus has been reached regarding the best methods.

**Conclusion:**

Measurement methods are expected to be standardized in the future to elucidate the skin mechanical properties of patients with lymphedema.

## 1 INTRODUCTION

Lymphedema is a common chronic disease characterized by localized tissue swelling owing to excessive lymphatic fluid retention in the interstitial compartment resulting from impaired lymphatic drainage.^1^ The pathophysiology remains largely undetermined. Skin conditions in patients with lymphedema have been identified in the International Society of Lymphedema (ISL) consensus staging system according to changes in skin mechanical properties such as hyperpigmentation, fat deposition, and warts, corresponding to the increasing severity of the disease stage.^2^ However, in the clinical practice of complex decongestive therapy for lymphedema, the assessment of skin mechanical properties is conducted subjectively by the evaluator through palpation.

The skin elasticity meter (Cutometer; Courage and Khazaka Electronic GmbH, Cologne, Germany) is a non‐invasive tool developed to perform objective quantitative measurements of skin mechanical properties.^3^ The measuring principle of this device is based on the suction method, where the skin's resistance to the negative pressure (firmness) and its ability to return to its original position (elasticity) are measured in real time and displayed as curves (penetration depth in mm/time). From these curves, various measurement parameters can be calculated related to the skin's mechanical properties, such as the elasticity and viscoelasticity of the skin surface. This device has demonstrated intra‐ and inter‐rater reliability in measuring the skin's mechanical properties on the upper and lower extremities of healthy individuals.^3^ Moreover, it has been applied in several studies within the cosmetic industry,^4^, ^5^ as well as in clinical settings for various skin diseases.^6^, ^7^, ^8^, ^9^

To date, the significance of skin elasticity measurement methods has received little attention despite the potential utility of the skin elasticity measurement device in evaluating the mechanical properties of the skin in patients with lymphedema. This article aims to provide a scoping review and offer an overview of studies that measure the skin mechanical properties of patients with lymphedema using a skin elasticity meter and discuss its potential applications in future clinical practice.

## 2 MATERIALS AND METHODS

### 2.1 Study design

This scoping review was conducted following the five‐stage framework initially presented by Arksey and O'Malley^10^ and subsequently refined by Levac, Colquhoun, and O'Brien.^11^ The study also adhered to the preferred reporting items for systematic reviews and meta‐analyses extension for scoping review (PRISMA‐ScR) guidelines.^12^, ^13^

### 2.2 Framework stage 1: Identifying the research question

We defined the research question as follows: “What studies have evaluated skin mechanical properties in patients with lymphedema using the skin elasticity meter?”

### 2.3 Framework stage 2: Identifying relevant studies

The search for articles was conducted on January 1, 2024. All articles were written in English and published through to the date of the search. The search strategy encompassed four electronic databases: MEDLINE, Cochrane Library, EMBASE, and CINAHL. In the database search, the key search concepts were categorized into four areas, namely, pathological condition, measurement device, skin condition, and measurement values. In the pathological condition section, one term was used: “lymphedema.” In the measurement device category, two terms were used: “skin elasticity meter” and “Cutometer.” In the skin condition category, four terms were used: “skin mechanical properties,” “mechanical properties of skin,” “elasticity,” and “distensibility.” In the measurement values category, three terms were used: “parameter,” “measurement,” and “outcome.” The Boolean operators “OR” and “AND” were used to link the search terms from each concept. A comprehensive list of key concepts and search terms is detailed in Table 1. Additional references were identified by manual searching.

**TABLE 1:** List of the key concepts and search terms.

Key concepts	No.	Search terms
Pathological condition	#1	lymphedema
Measurement device	#2	“skin elasticity meter”
	#3	Cutometer
	#4	(#2 OR #3)
Skin condition	#5	“skin mechanical properties”
	#6	“mechanical properties of skin”
	#7	elasticity
	#8	distensibility
	#9	(#5 OR #6 OR #7 OR #8)
Measurement values	#10	parameter
	#11	measurement
	#12	outcome
	#13	(#10 OR #11 OR #12)
Search formula	#14	#1 AND #4 AND #9 AND #13

The following criteria were used for inclusion in the study: (1) skin elasticity meter measurements for patients with lymphedema at any site of lymphedema; (2) articles published in English; and (3) original articles with a study design demonstrating a level of evidence higher than that typically associated with observational studies.

The exclusion criteria were as follows: (1) studies using a different Cutometer than the current model (owing to different measurement parameters); (2) articles published in languages other than English; (3) specific study designs, such as case reports, review articles, systematic reviews, and meta‐analyses; and (4) conference abstracts.

### 2.4 Framework stage 3: Study selection

Two independent reviewers rigorously evaluated the relevance of articles based on the predefined inclusion and exclusion criteria. In instances of disagreement, a third reviewer was consulted to achieve consensus on the inclusion of the articles. The initial screening involved reviewing the titles and abstracts of the articles retrieved. Subsequently, during the second screening, full texts of the articles deemed potentially eligible in the first screening were thoroughly reviewed to ascertain their suitability for inclusion in the study.

### 2.5 Framework stage 4: Charting the data

The reviewers collaboratively designed a data extraction scheme tailored to the objectives of the review and research question. The categories for data extraction included the first author's name, year of publication, title of the study, location of the study, study design, details of the subjects (number, age, cause of lymphedema, ISL classification, and duration of lymphedema), physical location affected (upper extremity or lower extremity), measurement site, probe diameter and suction negative pressure used, parameters measured in the study, and intended application of the device.

### 2.6 Framework stage 5: Collating, summarizing, and reporting the results

Data were meticulously extracted from all articles that met the eligibility criteria, followed by conducting numerical and thematic analyses. The findings from these analyses are presented in Table 2.

**TABLE 2:** Synthesis of eligible article characteristics.

					Subjects					Physical location				Parameters used in study						
No.	First author (year of publication)	Title	Study location	Study design	Number (female/male)	Age (mean ± SD)	Causes of lymphedema	ISL classification	Duration of lymphedema	Upper extremity	Lower extremity	Measurement site	Probe diameter used and suction negative pressure	R0	R2	R5	R6	R7	Other	Intended use of device
1	Hacard (2014)^14^	Measurement of skin thickness and skin elasticity to evaluate the effectiveness of intensive decongestive treatment in patients with lymphoedema: a prospective study	France	Before‐and‐after study	30 (24/6)	58.5 ± 14.6	Primary: 13 Secondary:17	I/II/III: 1/17/12	Median 11.5 (5−22)			+15 cm, −15 cm from the elbow Top of the hand +20 cm, −20 cm from the tip of the patella Top of the foot	6 mm 500 mbar		●	●	●			Intervention effect
2	Killaars (2015)^15^	Biomechanical properties of the skin in patients with breast cancer‐related lymphedema compared to healthy individuals	Netherlands	Case‐control study	18 (18/0)	63.0 ± 9.2	Breast cancer‐related lymphedema	–	–			Both lower arms, at the volar midpoint between the tip of the ulnar styloid process and medical epicondyle of the humerus	6 mm 450 mbar		●	●	●	●		Comparison with healthy individuals
3	Li (2018)^16^	Far‐infrared radiation thermotherapy improves tissue fibrosis in chronic extremity lymphedema	China	Before‐and‐after study	64 (−)	–	Primary: 15.6% Secondary: 81.3% Other: 3.1%	Late II/III: 40/24	–	〇 *n* = 18	〇 *n* = 46	Proximal third and distal third of the arm/thigh Proximal third and distal third of the forearm/leg Middle of the dorsum of hand/foot	6 mm 500 mbar	●	●	●			Q0	Intervention effect
4	Sano (2020)^17^	Development of a noninvasive skin evaluation method for lower limb lymphedema	Japan	Cross‐sectional study	25 (21/4)	64.0 ± 17.2	Primary: 7 Secondary: 18	I/II/III: 14/19/12	–		〇	Thigh at four points: anterior, posterior, medial, and lateral (the average values of bilateral forearms measured for predictive value calculated)	–		●	*Listed under another name				Development of measurement methods

*Note*: –, data not shown.

### 2.7 Ethical statement

The authors’ institutions have confirmed that ethics committee approval was not required for this study because it was not a study on human subjects.

## 3 RESULTS

From a comprehensive search across all sources, 621 results were obtained. After the exclusion of 56 duplicate articles, 565 articles remained for eligibility screening. Upon screening titles and abstracts, 560 articles were further excluded. The full texts of the remaining five articles were thoroughly examined for eligibility, leading to the exclusion of one article. Finally, four eligible articles^14^, ^15^, ^16^, ^17^ were included in this study. Manual searching did not yield any additional eligible articles. The process of article review, selection, and eligibility assessment at each stage is depicted in the PRISMA flow diagram^12^, ^13^ (Figure 1).

**FIGURE 1:** PRISMA flow diagram.

### 3.1 Synthesis of eligible article characteristics

Table 2 provides a summary of the characteristics of the eligible articles. All articles included in this review were published after 2010 and originated in France, the Netherlands, China, or Japan. The study designs comprised two cross‐sectional studies and two before‐and‐after studies. In total, 137 patients with lymphedema, predominantly secondary lymphedema, were encompassed in this review. In addition, none of the studies observed patients with ulceration, and only lymphedema was included. Regarding the physical location, three articles addressed both the upper and lower extremities. Measurement sites were not standardized and set individually by each study. In the articles mentioned, the probe diameter was 6 mm, and the suction negative pressure was 450−500 mbar. The parameters investigated included R0, R2, R5, R6, R7, and Q0, with the parameter R2 being utilized across all studies. The intended application of the device was the intervention effect (*n* = 2), comparison with healthy individuals, and the development of measurement methods.

## 4 DISCUSSION

We conducted a scoping review to ascertain “What studies have evaluated mechanical properties of skin in patients with lymphedema using the skin elasticity meter?” Four articles satisfied the inclusion criteria. Here, we offer an overview constructed from the current perspectives and insights derived from these findings.

Our review of the available literature indicates that the investigation into the mechanical properties of skin in patients with lymphedema, facilitated by the skin elasticity meter, represents a recent interest within the field, as evidenced by the growing number of reports since the 2010s. These studies have been conducted worldwide, in both developed and emerging nations, likely reflecting the importance of discerning the mechanical properties of skin in patients with lymphedema and providing an objective metric to evaluate the efficacy of treatment modalities. However, the inclusion of only four articles highlights the early stage of research in this area. In the four articles, several commonalities were observed. The used parameters included R0 (distensibility), R2 (gross elasticity), R5 (net elasticity), R6 (viscoelasticity), and R7 (biological elasticity),^3^ with R2 being employed in all studies to denote the resistance to mechanical force versus the ability for time‐delayed recovery. The consistent use and endorsement of the R2 parameter across various studies highlights its potential applicability for patients with lymphedema^18^, ^19^, ^20^; nonetheless, its utilization remains a topic for further discussion.

On the other hand, four articles in this review were not standardized in their measurement methods, such as the causes of lymphedema (primary and/or secondary), stage of ISL classification, measurement sites, and using parameter combinations. Therefore, at present, there are significant challenges in the comparisons and generalization among these studies. In the future, it is necessary to establish a standardized measurement methodologies for patients with lymphedema using skin elasticity meter device, as the number of study reports increases.

The application of skin elasticity meters for measuring skin mechanical properties has been insufficiently addressed in the literature for an extended period despite its demonstrated value in diverse fields, particularly in clinical medicine.^6^, ^7^, ^8^, ^9^ The predominance of palpatory assessments, such as “pitting edema,”^21^ in the clinical management of lymphedema, may account for the limited use of skin elasticity meters for assessing skin mechanical properties in patients with lymphedema. Currently, a standardized protocol for objective measurement does not exist. Although ultrasound has been employed to evaluate skin conditions in patients with lymphedema,^22^, ^23^ it predominantly measures subcutaneous stiffness rather than specific skin mechanical properties, thus not aligning with ISL classification stages. Consequently, an immediate necessity is to establish a measurement methodology using skin elasticity meters, and an increase in scholarly contributions is anticipated. Moreover, the cost implications of acquiring such devices may restrict their broad application, particularly in developing countries where lymphatic filariasis‐induced lymphedema is common, and financial or environmental limitations may preclude measurement efforts. Research initiated in the 2010s and continuing to date is anticipated to lead to global standardization, contributing to the elucidation of skin mechanical properties and the development of therapeutic strategies for patients with lymphedema.

This study had several limitations, including a database search limited to publications up to January 1, 2024, thereby excluding articles published subsequently as well as non‐English articles, gray literature, and prior review articles. Moreover, the assessment of the efficacy of using skin elasticity meters in patients with lymphedema was not conducted, as per the discretion allowed in the PRISMA‐ScR guidelines.^12^, ^13^ This approach reflects the nature of scoping studies, which do not evaluate the quality of evidence; thus, such studies are unable to determine the robustness or generalizability of the findings.

## 5 CONCLUSION

This review summarized the examination of skin mechanical properties in patients with lymphedema utilizing the skin elasticity meter. Given the escalating interest in this research domain since the 2010s, a consensus on the optimal measurement methodology remains elusive. Nonetheless, this approach has the potential to emerge as a prevalent measurement technique in the future. An increase in scholarly reports and a convergence toward standardized measurement methodologies are anticipated.

## CONFLICT OF INTEREST STATEMENT

The authors report no conflicts of interest.

## Data Availability

Data are available upon reasonable request from the corresponding author.
